The article "Innovation of Network Political and Ideological Education in Colleges Based on Service Concept in Network Environment" was retracted in 2023. Reasons: signs of a paper mill; suspected computer-generated content; unreliable results or conclusions; concerns about the data.

# Innovation of Network Political and Ideological Education in Colleges Based on Service Concept in Network Environment

**DOI:** 10.1155/2022/2564447

**Published:** 2022-08-18

**Authors:** Doudou Yin

**Affiliations:** School of Marxism, Shanghai Civil Aviation College, Shanghai 200232, China

## Abstract

With the ongoing advancement of information technology, we must adopt the proper mindset when addressing the opportunities and difficulties that political thought education in institutions of higher learning face in the current network environment, take full advantage of the network's benefits, and take proactive steps to address the innovation of political thought education in institutions of higher education under the network environment. Based on the field of political thought education itself, this article studies the new characteristics of political thought education communication in institutions of higher learning under the network environment, analyses the problems and causes in the process of political thought education innovation in institutions of higher learning under the network environment, and explores a number of measures to improve the innovation level of political thought education under the network environment. This article describes the significance, traits, and internal connections between network media and the innovative development of political thought education in higher education institutions and proposes a cutting-edge course for the advancement of political thought education in higher education in the network era. In parallel, a system for early detection and evaluation of political thought education in higher education institutions is being built. The accuracy of this algorithm, according to experiments, can reach a high level of 95.31%, which is impressive. This study has served as a guide and a source of encouragement for institutions of higher learning to use network carriers to deliver political thought education.

## 1. Introduction

The way people live, think, and value has changed as a result of the network. With the advancement and transformation of the times, new research into the dissemination of political thought education is required [1]. The rapid development of networks has also changed higher education institutions' approaches to teaching political thought. Institutions of higher learning are inevitably influenced by the network information society with the constant demand for information development as a place to develop high-quality talents. Higher education institutions are now the primary incubators for in-depth Internet application development. Political thought education in higher education institutions plays a significant role in the background of young college students' lives, and it is directly related to how smoothly new college students adjust to their new environment [2]. The network's use in various fields of study not only advances those fields as a whole but also improves the network's capabilities. The network environment is currently understood in academic circles in both broad and specific ways. The former is used in the sense of the “network age,” which alludes to the modern social landscape. The latter refers to the virtual environment, which is the cyberspace to be socialised [3]. Political thought education, or the cultural transmission of an ideology, dulls people and gives them a sense of being removed from reality when it is taught using the traditional educational model. The learning demands of contemporary students in a network environment cannot be met by traditional political thought education practices. Due to the proliferation of media outlets in recent years, many things that are done to increase ratings and clicks frequently violate social morality [4]. Political thought education, which disseminates information through traditional media, is significantly less effective when impacted and influenced by the network. In light of this circumstance, a network and political thought education are essential. In the new era, it is difficult and urgent to figure out how to use network carriers to innovate political thought education in institutions of higher learning and how to view the network as a key position of political thought education in such institutions.

The article "Innovation of Network Political and Ideological Education in Colleges Based on Service Concept in Network Environment" was retracted in 2023. Reasons: signs of a paper mill; suspected computer-generated content; unreliable results or conclusions; concerns about the data.

The traditional methods of educating people about political thought must be greatly modified because of the numerous changes brought about by the Internet [5]. Due to its strong informational efficacy, limitless information transmission, vast amount of information, and prompt two-way communication, Internet information has a very broad audience [6]. The information society is a totally unrestricted environment. The information that students need in the network age is much more detailed and extensive than what they receive in the classroom. This proposes new standards for political thought education in higher education institutions in a network environment [7]. We need to do a good job of innovating political thought education for college students under the network environment in order to deal with the new environment and new tasks. The openness of the network's political thought education environment; how to effectively and correctly teach students to use the network to choose useful information; and how to create a trinity education model that balances the needs of the family, society, and school are all pressing problems that need to be addressed right now. This article analyses the innovation of network political thought education in higher education institutions based on the service concept. The innovations of this article are as follows:

1. This article analyses the innovation of political thought education in institutions of higher learning based on the development and change of the network environment and firmly grasps the pulse of the times against the background of the interactive development of social network and culture. This article compares the pertinent theories and methodologies while also understanding the opportunities and difficulties that the innovation of political thought education in institutions of higher learning under the network environment faced in the new period. This understanding is followed by an analysis of potential countermeasures for the innovation of political thought education in institutions of higher education under the network environment.
2. The concept, content, carrier, and mechanism of political education in this article and the main path of “how to innovate” are explored, and the innovative development of political thought education in institutions of higher learning is profoundly explained, with a comprehensive and systematic view. In addition, this article starts with the various factors that affect the communication effect and then explores the countermeasures of network innovation of political thought education on this basis, hoping to provide a reference for the practice.

The article "Innovation of Network Political and Ideological Education in Colleges Based on Service Concept in Network Environment" was retracted in 2023. Reasons: signs of a paper mill; suspected computer-generated content; unreliable results or conclusions; concerns about the data.

## 2. Related Works

The rapid development of information technology has greatly changed the environment of college students' political thought education; seriously affected a series of problems such as traditional ways, methods, and contents of political thought education; and brought brand-new opportunities and many challenges to political thought education in institutions of higher learning. Therefore, in recent years, many experts, scholars, and political thought educators have begun to think about political thought education in institutions of higher learning under the background of network media and have made some preliminary research results.

Porcello and others believed that the Internet has enriched ideological and political education resources, broadened the means of ideological and political education, and broke through the limitations of time and space, but to a certain extent, it has brought challenges to the content, methods, and means of ideological and political education and the quality of teachers [8]. Su pointed out that the characteristics of network communication include: the timeliness of the communication speed, the openness of the communication range, the mass of the communication content, the interaction of the transmission and reception relationship, the virtuality of the communication environment, and the comprehensive type of communication form [9]. Cusumano analysed and explored the impact of media changes and media environment changes on the innovation and development of ideological and political education in colleges and universities through a comparative analysis of the research results of media development and innovation in the fields of communication and journalism. The bottleneck restriction and innovative path provide theoretical support and practical support [10]. Weld et al. comprehensively described the current situation of network ideological and political education research as well as the theoretical basis of network ideological and political education research. At the same time, in-depth research and innovation are carried out on the relationship between the Internet and ideological and political education, the nature and characteristics of Internet and ideological and political education, the formation and development of Internet ideological and political education, and the function and value, management and development of Internet ideological and political education [11]. Han and others believed that the purpose of research on ideological and political education of college students in the network environment is to grasp the laws of network communication and innovate the methods and content of ideological and political education in colleges and universities [12]. Emanuel et al. believe that in the network environment, the political concept of college students is weak, and the ideological concept is eroded to a certain extent, so the ideological and political education work in the network environment has a certain significance [13]. Srivastava et al systematically discussed the opportunities and challenges brought by the network environment to ideological and political education in colleges and universities and focused on the countermeasures and measures to strengthen ideological and political education of college students in the network environment [14]. Castle et al. believed that the network environment expands the subject and object of ideological and political education and also broadens the carrier and the circle, but to a certain extent; it also challenges the authority of teachers and confuses the choice of students' information [15]. Paden studied the current situation of the ideological and political education function of college network culture, analysed the problems existing in the realisation of the function of network culture ideological and political education in colleges and universities, and put forward corresponding countermeasures [16]. According to the technical difficulties of the media itself and the practical application dilemma in the innovation and development of ideological and political education in colleges and universities, Hovsepian analysed the media's assistance in the innovation and development of ideological and political education in colleges and universities from the perspectives of educational subject and object, educational content, educational carrier, and working mechanism [17].

The article "Innovation of Network Political and Ideological Education in Colleges Based on Service Concept in Network Environment" was retracted in 2023. Reasons: signs of a paper mill; suspected computer-generated content; unreliable results or conclusions; concerns about the data.

This article analyses the innovation of political thought education in institutions of higher learning based on a thorough analysis of pertinent literature and the service concept. This article compares relevant theories and methodologies based on a literature review, grasps the opportunities and difficulties faced by the innovation of political thought education in higher education institutions under the network environment in the new period, and then proceeds to a countermeasure analysis of the innovation of political thought education in higher education institutions under the network environment. In parallel, a system for early detection and evaluation of political thought education in higher education institutions is being built. The performance of this algorithm is very high, according to experiments. The author hopes that this research will be able to offer some recommendations for the modernisation of political thought instruction in higher education institutions.

## 3. Methodology

### 3.1. Network Media and Innovative Development of Political Thought Education

Nowadays, a series of emerging network media are increasingly affecting people's lives. The emergence of the Internet marks that the combination of information technology and communication technology has reached a brand-new level, increasingly enriching people's lives, and providing people with a borderless and equal exchange stage [18]. It has the following characteristics: (1) virtuality, (2) openness, (3) interaction, and (4) timeliness. Internet has increasingly exerted a wide and profound influence on college students' political thought education. In this environment, political thought education of college students is bound to face opportunities and challenges brought by new technologies. Nowadays, the content and traditional communication means of political thought education can no longer meet the needs of college students, and the traditional theoretical indoctrination conflicts with the open network communication environment. Under the influence of the network environment, the information transmitted by books, television, and classrooms is questioned by students [19]. Actually, network political thought education has two connotations: one is political thought education under the network environment, and the other is political thought education based on the network. The former is a broad understanding of network political thought education, and the latter is a narrow understanding of network political thought education. As for political thought education of a special communication activity, it is included in the general communication concept. Political thought education is a kind of communication activity, but compared with the general communication, the communication of political thought education focuses more on the research of the content, objectives, and elements of communication. Political thought education is closely related to network communication. On the one hand, network is the new environment and carrier of political thought education in institutions of higher learning. Therefore, the need for discipline construction of political thought education in institutions of higher learning and the requirement of adapting to the development of the times make political thought education in institutions of higher learning have to do a good job in network communication. On the other hand, political thought education itself is a special form of communication activities, so its expression and related skills can guide the development of political thought education. The relationship of communication elements of political thought education under the network environment is shown in Figure 1.

The article "Innovation of Network Political and Ideological Education in Colleges Based on Service Concept in Network Environment" was retracted in 2023. Reasons: signs of a paper mill; suspected computer-generated content; unreliable results or conclusions; concerns about the data.

Diversification, differentiation, and integration are the characteristics of the innovation of political thought education carriers in institutions of higher learning. The varied features include: the traditional curriculum carrier using the classroom as the primary channel, the campus paper media carrier, the carrier of campus cultural activities in various forms, and the carrier of new media communication represented by the Internet and mobile terminals. The management carriers of various organisations and management departments, various types of relationship carriers, etc., are also present at the same time and exhibit the development trend of a hundred flowers blooming. Users of networks receive a personalised experience thanks to network communication. The characteristics of network communication demonstrate that it has significant advantages over traditional media as a vehicle for the dissemination of political thought education [20]. Political thought education is no exception to the long-standing legacy of conventional educational techniques and approaches in textbooks, teachers' words, and actions. The expansion of network technology has increased both the quantity and speed of information transfer, greatly expanding people's horizons. Traditional methods of knowledge dissemination fall short in comparison to the global openness and sharing of information. Political thought education has a significant and widespread impact on the Internet. All-media was founded on the idea of adapting to social advancement and technological advancement. It was proposed in light of the integration and coexistence of old media, dominated by paper, new media, carried by mobile phones and the Internet, and modern media, dominated by television and radio. It dynamically described all the current forms of communication in addition to including all-media. A two-way conversation between the subject and the object of education via the Internet takes place during the process of educating people about political thought. It describes a collaborative relationship between the subject and the educational target in a particular setting that acknowledges ideas, information, and feelings. It not only challenges the established and conventional position of academics and well-educated individuals, but it also represents the possibility of dialogue on an equal footing.  Figure 2 shows the proportion of Internet users of different ages in 2015.

The article "Innovation of Network Political and Ideological Education in Colleges Based on Service Concept in Network Environment" was retracted in 2023. Reasons: signs of a paper mill; suspected computer-generated content; unreliable results or conclusions; concerns about the data.

The innovative development of political thought education in institutions of higher learning and the whole media are a long-term relationship of mutual benefit, mutual promotion, and common progress. Their development ideas are consistent. The development content has certain compatibility. The dissemination process of political thought education in institutions of higher learning under the network environment refers to a series of political thought education activities carried out on the platform of network media. The main content of the study is the correlation and interaction of information sending, receiving, and feedback, so any problem in any stage will affect the final effect of political thought education communication. The new ideas and viewpoints of political thought education in institutions of higher learning fit perfectly with the actual needs of the all-media era and have a better development opportunity in the all-media era. Network political thought is not only ideological and moral education, but also the organic unity of various elements. Among them, political education and ideological education are the direction and soul, moral education and law and discipline education are the key points, and mental health education is the foundation. All aspects cannot be separated, let alone replaced by each other. The network environment is organically combined with political thought education, and the network environment makes it possible to carry out political thought education with the help of the network, providing the premise and foundation for it. At the same time, as a new tool and channel for political thought education, the network has greatly promoted the comprehensive reform of political thought education concept, content, ways, and methods under the network environment. The innovation and development of political thought education in institutions of higher learning has entered a new development period, showing the following new features: (1) The times: the innovative development of political thought education in institutions of higher learning has strong characteristics of the times. (2) Humanity: the essence of socialism is to realise the all-round development of people. (3) Innovation: the innovation of political thought education in institutions of higher learning is mainly reflected in its content, concept, carrier, and working mechanism.

The article "Innovation of Network Political and Ideological Education in Colleges Based on Service Concept in Network Environment" was retracted in 2023. Reasons: signs of a paper mill; suspected computer-generated content; unreliable results or conclusions; concerns about the data.

### 3.2. Innovative Strategy of Network Political Thought Education in Institutions of Higher Learning Based on Service Concept

Under the network environment, the improvement and innovation of college students' political thought education is an important part of political thought education's own development and perfection. To solve the complicated contradictions and successfully complete the tasks and objectives of political thought education, we should not only adhere to theoretical guidance, but also require political thought education subjects to correctly grasp and apply the principles of network political thought education. With the support of network technology, the spread of knowledge and ideas has the advantages of wide coverage and high speed. First, it can make political thought education be carried out longer and wider without the limitation of time and scope. Second, the educated are also not limited by time, region, and nature of work, so they can receive better political thought education anytime and anywhere. The innovative principles of political thought education in institutions of higher learning under the network environment are as follows: (1) people-oriented principle, (2) creative principle, (3) initiative principle, and (4) systematic principle. By developing thematic websites and other tools to provide rich and colourful content and flexible information communication mode, educators of political thought education in institutions of higher learning can easily draw college students to the network. This is made possible by the inclusive content of network information, the interactive communication mode, and the high timeliness of information. In cyberspace, people communicate, share knowledge, and advance together. In addition, it is important to align development law with the specific requirements of college students' success and growth, as well as adjust to the broader goals of higher education reform and innovation. First and foremost, we can establish a special campus network management department and strictly draught the necessary network code of conduct while using scientific methods to manage effectively in accordance with the law. Second, institutions of higher education should create online communities that are tailored to the needs and characteristics of their students, support their right to voice their opinions on current events, and regularly publish material that is pertinent to students.  Table 1 displays the educational levels of Chinese Internet users in 2015 along with the methods used by college students to find information.

The article "Innovation of Network Political and Ideological Education in Colleges Based on Service Concept in Network Environment" was retracted in 2023. Reasons: signs of a paper mill; suspected computer-generated content; unreliable results or conclusions; concerns about the data.

It is clear that there is a growing connection between college students and the Internet, and that the Internet has a significant impact on every aspect of students' lives. Political thought education has interactive effects in the network era, and those who receive it can actively choose what information they want to learn rather than passively taking it in. Higher education institutions should rely on the network carrier to create a strong sense of learning, carve out a distinct Marxist theoretical education position online, and use positive and healthy thoughts as a guide. They should also open up various columns of political thought education with cutting-edge theories and occupy network positions. Modern college students have a free space for their growth because they are a group with a strong sense of autonomy and a flamboyant personality. Students have the freedom to learn, have fun, browse information, and download materials at any time as they please. They can also select different types of online content based on their interests, which creates room for the development of students' subjective consciousness. The educated's mental state is actively generated and constructed by them rather than being shaped by outside forces. There is no way to achieve the process of the educated internalising political thought education through coercive measures. The most crucial educational strategy that teachers should master is entertainment. We can only get good results if we make education more appealing. Political thought education's inherent lack of attractiveness is determined by its own characteristics. The growth of the Internet has given rise to more multimedia technologies, which can display the engaging educational material through text, sounds, videos, animations, and other means. This has made education less dull and increased the appeal of the political thought education material. Educators need to position themselves correctly, not in a high position, and should discuss and learn from the educated. At the same time, educators need to consider the specific characteristics of the educated, and when carrying out political thought education, they should meet each other's needs and start from each other's interests, so as to improve the effect of political thought education.

The article "Innovation of Network Political and Ideological Education in Colleges Based on Service Concept in Network Environment" was retracted in 2023. Reasons: signs of a paper mill; suspected computer-generated content; unreliable results or conclusions; concerns about the data.

The only way for institutions of higher learning to increase the influence and attraction of educational carriers, while simultaneously meeting the multilevel and individualised needs of college students, is by “fully grasping the trend and law of media convergence and development,” occupying the network position of mainstream ideology, and innovating educational carriers and methods. Higher education institutions may also regularly engage in online reading and storytelling activities, which not only satisfy students' thirst for knowledge but also increase their knowledge stores through communication. These activities help students develop a positive outlook on life and strong cultural literacy while also enhancing their independence and creativity. The use of network information technology in scientific research and teaching has become a necessary component of educational modernisation. Higher education institutions should make the best use of current network technology to build digital libraries, offer college students rich online courses, and give students access to online course options, video open classes, and online learning-quality courses. Under the modern environment, it is required that the network political thought education environment should not stick to the old routine; break the tradition of sticking to the classroom and classroom space; and extend the classroom to the school's electronic reading room, dormitory, and even the family.

## 4. Innovation Evaluation and Early Warning System Construction of Political Thought Education in Institutions of Higher Learning

In higher education institutions, political thought education is a crucial component of developing top-tier talent for the twenty-first century. Its evaluation criteria ought to establish a scientific procedure and serve as a benchmark for political thought instruction. The gathering, assembling, and analysis of information is essentially the goal of evaluation. At this point, the evaluation work primarily makes use of contemporary evaluation methods and techniques to gather and compile all required evaluation data. After this type of information's accuracy and dependability are established, a valuable judgement is produced by combining qualitative and quantitative evaluation objects to create the evaluation result. Evaluations of education should adhere to the values of fairness, accuracy, efficacy, and modernity. To ensure that the system can contribute to the long-term development of education and beneficial guidance for teaching and learning, it should ensure the universality and scientificity of the evaluation system as well as the authenticity and clarity of the evaluation process. Because some attribute values are frequently vacant in real-world databases for a variety of reasons, those data have little bearing on the knowledge discovery process. Frequency statistics can be used to address data defects if the types of defects fall under discrete continuous attributes and discrete attributes.

The article "Innovation of Network Political and Ideological Education in Colleges Based on Service Concept in Network Environment" was retracted in 2023. Reasons: signs of a paper mill; suspected computer-generated content; unreliable results or conclusions; concerns about the data.

Firstly, the candidate word set is initialised, and the current test data are calculated by the *δ*−*ε* algorithm:

(1) $$\begin{array}{c} i_{1}\leq i_{2}\leq \ldots \leq i_{N},\;\varepsilon_{1}\left(i,j\right),\delta_{1}\left(i,j\right). \end{array}$$

Thereafter, the HMM parameter *λ*^*∗*^ is revalued with *δ*_1_(*i*, *j*). Let the HMM parameter of the trained candidate word set be *λ*:

(2) $$\begin{array}{c} \left\{if\left(\lambda >\lambda^{*}\right),V=V-\upsilon_{\lambda^{*}}\right\}\text{until}\left(\text{all}\lambda <\lambda^{*}\right). \end{array}$$

A new candidate word set *V*^*∗*^=*V* is obtained. *D*(*n*, *m*) is set as the cumulative DTW distance from the (*n*, *m*) partial path:

(3) $$\begin{array}{c} D\left(n_{i},m_{i}\right)=d\left(n_{i},m_{i}\right)+A,\\ A=\min\left\{D\left(n_{i-1},m_{i-1}-1\right),D\left(n_{i-1},m_{i-1}-2\right),D\left(n_{i-1},m_{i-1}\right)\right\},\\ D\left(n_{i},m_{i}\right)=d\left(n_{i},m_{i}\right)+B,\\ B=\min\left\{D\left(n_{i-1},m_{i-1}-1\right),D\left(n_{i-1},m_{i-1}-2\right)\right\}. \end{array}$$

A training sample *i*_*t*_ is randomly selected in the hyperplane constrained space. Among them, *i* represents the intrinsic property of the sample, and *t* represents the extrinsic activity of the sample, which is brought into the formula:

(4) $$\begin{array}{c} f\left(\omega ,i_{t}\right)=\frac{\lambda }{2}{\left\|\omega \right\|}^{2}+l\left(\omega ,\left(x_{i_{i}},y_{i_{t}}\right)\right). \end{array}$$

Subgradient solution to the formula is as follows:

(5) $$\begin{array}{c} \nabla_{t}=\lambda \omega_{t}-I\left\lfloor y_{i_{t}}\left\{\omega_{t},x_{i_{i}}\right\}<1\right\rfloor y_{i_{t}}x_{i_{i}}. \end{array}$$

where *I*⌊*y*_*i*_*t*__{*ω*_*t*_, *x*_*i*_*i*__} < 1⌋ is the indicator function, the value range is two values; if it is true, it is 1, otherwise it is 0. Inputting the user interest point data set *S*, the regularisation factor *λ*, and the sample external activity *T*, the iteration of one cycle can be expressed as:

(6) $$\begin{array}{c} \omega_{t+1}\leq \omega_{t}-\beta_{t}\nabla_{t} \end{array}$$

where *β*_*t*_=1/*λ*_*t*_ is the adaptive step size factor, which is negatively correlated with the number of iterations. The cumulative distance *D*(*n*_*i*_, *n*_*i*−1_) is calculated based on the DTW search strategy of the test data itself and converted it into fuzzy closeness, and the following formula is used to calculate the result of the Viterbi algorithm:

(7) $$\begin{array}{c} d_{t}\left(j\right)=\underset{1\Gamma t\Gamma N}{\max}\left\lfloor d_{t-1}\left(i\right)a_{ij}\right\rfloor b_{j}\left(O_{t}\right). \end{array}$$

Process simulation and process improvement are applications such as workflow management, which can be divided into three stages. The process or optimisation of process modeling is a clear representation and a formal method with different levels of abstraction. Process analysis and reliable model are the foundation, and process simulation is to find out and provide guidance. Their seamless connection is the key factor that affects the performance of the workflow model, but these three stages are constantly evolving, but there are also major problems such as traditional process modeling and simulation process integration. In this article, the data mining method is used to screen evaluation indexes, which can quickly and efficiently mine massive text information and then process and analyse it. This model analyses the word frequency of relevant authoritative literature and screens out the evaluation indexes to be analysed. The indicators of the evaluation system are shown in Table 2.

The article "Innovation of Network Political and Ideological Education in Colleges Based on Service Concept in Network Environment" was retracted in 2023. Reasons: signs of a paper mill; suspected computer-generated content; unreliable results or conclusions; concerns about the data.

In order to further make a comprehensive fuzzy evaluation on the quantitative data of users' invisible warning, it is integrated into the decision analysis system and mechanism. The overall design structure of the system is shown in Figure 3.

The influence of dimensions should be removed and the original data should be standardised when thoroughly analysing the data of the index system. The following are the steps in the data standardisation processing: first, the index's negative value that has a negative impact on the evaluation's outcome is taken; second, the following formula is used for dimensionless, or standardised, processing of index data. The primary objective of the submodule of political thought education effect analysis is to assess the multifaceted effects of the customised political thought education programme created by the political thought education implementation submodule. In order to provide data export and printout functions, a comprehensive data query refers to the querying of a variety of business information produced by the evaluation of administrators or office staff. Department heads or administrators may request student evaluations and processing for some query results, and teachers teaching the same class within the department may take course materials. The dynamic warning submodule of political thought education primarily realises the early detection of students with risky thoughts and provides warning advice as well as timely active intervention measures. It ensures the smooth development of the overall national security concept and provides a solid foundation for students' healthy development by paying attention to their psychological traits.

## 5. Experimental Analysis

Although political thought education is a continuous dynamic process, some standard values may be different from reality, but it has been proved to be ideal in practice, thus reflecting the characteristics of development in the static indicators. The preprocessing process includes word segmentation, stop words removal, and semantic feature extraction [21]. The most important part of word segmentation is the selection of dictionaries. In order to avoid the problems caused by the limitations of dictionaries, this model scans Chinese phrases in word segmentation dictionaries based on prefix dictionaries to achieve efficient word graph scanning and generate directed acyclic graphs. The running environment needs to support the running machine environment above WIN2000. For higher-level operating systems, the software can be further maintained to achieve its stability. The final simulation result is shown in Figure 4.

In order to make the test data set provided by the Sklearn database more appropriate to the dynamic early warning model of political thought education, the regression mapping process is carried out on the data set of user behavior and the data set of user invisible points of interest. The index selected in this article not only reflects the main characteristics of the quantitative object of the subsystem but also helps other subsystems. Although the selected index factor is representative, it cannot fully reflect the information to be expressed. The simulation diagram of decision analysis effect of the standard fuzzy neural network algorithm is shown in Figure 5.

Data conversion and transmission time: the registration of students and the recitation and conversion time of teachers' evaluation results can be set reasonably so that it will not affect users' use, and the key is to meet users' needs. In Simulink, the visual interface is used to view and edit various parameters of the network, such as weight, offset vector, and activation function. Adjusting the weight of the network can make the error between the network output and the expected output smaller. Simulation of decision analysis effect of improved fuzzy neural network algorithm is shown in Figure 6.

The article "Innovation of Network Political and Ideological Education in Colleges Based on Service Concept in Network Environment" was retracted in 2023. Reasons: signs of a paper mill; suspected computer-generated content; unreliable results or conclusions; concerns about the data.

It can be seen that the actual working effect of the dynamic early warning model of political thought education has been greatly improved by introducing the separation factor of hot and cold data, the random gradient descending factor, and the decision analysis system. A comparison of evaluation results of different algorithms is shown in Figure 7.

It can be seen that the accuracy of this evaluation method is as high as 95.31%, which is a high level. Considering that the input data in the actual application process generally conform to the specific structural characteristics, it is considered that this method has certain reliability in the evaluation of political thought education in institutions of higher learning, and the calculation is simple and fast.

## 6. Conclusions

Since the advent of information technology, the network has had a distinctive impact on all facets of human existence. The new era introduces new goals and specifications for political thought education in institutions of higher learning and embarks on a new journey for political thought education. As a requirement of the network era, political thought educators in higher education institutions in the new era should fully implement the scientific concept of development and work to innovate political thought education for college students under the new situation. The innovation and advancement of political thought education in higher education institutions should be in line with the progress of the new era. Through political thought education communication activities, college students can internalise the transmitted information in their hearts and externalise it in their actions, which is a sign that political thought education communication in institutions of higher learning is effective. The form and content of political thought education in higher education institutions should be improved. The main melody should serve as our guide, and we should not only use network communication to “set the agenda,” but we should also innovate the format of network political thought education and fully exploit its potential. This article aims to synthesise the flaws in the innovation and development of political thought education in institutions of higher learning, analyse the opportunities and problems it faces in the network media era, and offer some recommendations and approaches for its innovative development in the all-media era. This article also develops a system for monitoring and assessing political thought education provided in higher education institutions. The accuracy of this algorithm, according to experiments, is at a high level, reaching up to 95.31%. The innovation of political thought education in higher education institutions is crucial in the network environment. Another significant task given to us in the new era is to strengthen the research on college students' political thought education in a network environment. We will come up with a better solution to the issue when we adjust our thinking and the environment. We can only provide the theoretical and technical support for the discipline development of network political thought education in institutions of higher learning in the new era by closely following the trend of the times and fully utilising the benefits of network information technology.

The article "Innovation of Network Political and Ideological Education in Colleges Based on Service Concept in Network Environment" was retracted in 2023. Reasons: signs of a paper mill; suspected computer-generated content; unreliable results or conclusions; concerns about the data.

## Figures and Tables

**Figure 1:** Relationship diagram of communication elements of political thought education under the network environment.

**Figure 2:** Proportion of Internet users of different ages.

**Figure 3:** Overall design structure diagram of the system.

**Figure 4:** Simulation diagram of dynamic early warning model of political thought education based on standard SVM algorithm.

**Figure 5:** Simulation diagram of decision analysis effect of standard fuzzy neural network algorithm.

**Figure 6:** Simulation diagram of decision analysis effect of improved fuzzy neural network algorithm.

**Figure 7:** Comparison of evaluation results.

**Table 1:** Proportion of Chinese netizens with different educational levels and ways for college students to obtain information.

Academic degree	Proportion (%)	Access to information	Proportion (%)
Primary school and below	9.15	Network	72.14
Junior school	23.14	Books and magazines	15.02
Senior high school	38.46	Broadcast	3.15
Universities and colleges	16.89	TV	8.67
Bachelor's degree or above	12.36	Other	1.02

**Table 2:** Evaluation of each index of the system.

	Primary index	Secondary index
Evaluation index system	Model of instruction	Theme demonstration education
		Party lesson education
	Body scale	Participation ratio of social evaluation
		Student evaluation of teaching
	Learning content	Patriotic education
		Integrity education
		Discipline education
	Hard score	Relevant recognition
		Number of critical reports
		Innovation ability
	Learning performance	Activity participation
		Preparation before class

## Data Availability

The data that support the findings of this study are available from the corresponding author upon request.
